# Biomedical Application of Identified Biomarkers Gene Expression Based Early Diagnosis and Detection in Cervical Cancer with Modified Probabilistic Neural Network

**DOI:** 10.1155/2022/4946154

**Published:** 2022-09-10

**Authors:** K. Ramesh, Pankaj Agarwal, Vandana Ahuja, Bilal Ahmed Mir, Shvets Yuriy, Majid Altuwairiqi, Stephen Jeswinde Nuagah

**Affiliations:** ^1^Head of the Department, PG & Research Department of Computer Science and Applications, Vivekanandha College of Arts and Sciences for Women (Autonomous) Elayampalayam, Tiruchengode, Tamilnadu, India; ^2^School of Engineering and Technology, K.R. Mangalam University, Gurugram, Haryana, India; ^3^Department of Computer Science and Engineering, Swami Vivekanand Institute of Engineering and Technology, Ramnagar, Banur, Punjab, India; ^4^Graduate School of Science and Engineering for Education, University of Toyama, Toyama, Japan; ^5^Institute of Control of Science V.A. Trapeznikov RAS, Financial University Under the Government of Russian Federation, Russian Federation, Moscow, Russia; ^6^Department of Computer Science, College of Computers and Information Technology, Taif University, Taif, Saudi Arabia; ^7^Department of Electrical Engineering, Tamale Technical University, Tamale, Ghana

## Abstract

Cervical squamous cell carcinoma (CSC) is expected to rise to become the fourth most prevalent cancer in women globally and to replace breast cancer as the top cause of death in women in the future years, according to the World Health Organization. According to the World Health Organization, developing countries are responsible for 86 percent of all cervical cancer cases globally in women aged 15 to 44 (WHO). Cancer mortality is associated with the largest amount of monotonous antecedent in low- and middle-income nations, while cancer mortality is associated with the least amount of monotonous antecedent in high-income countries. Cervical cancer is thought to be caused by aberrant proliferation of cells in the cervix that is capable of stealing or invading other human organs, according to current thinking. Cancer of the cerebral cell is the most prevalent kind of cancer in women. It is expected that cervical squamous cell carcinoma (CSC) will be the fourth most frequent cancer in the world and the main cause of death in women by the year 2050. Despite the fact that technology has improved tremendously since then, this is still the case. When compared to high-income countries, low- and middle-income countries have the highest consistent antecedent for cancer mortality, according to the World Cancer Research Fund. Cancerous growths of cells in the cervix, such as cervical cancer, are caused by cells that have the ability to steal from or invade auxiliary organs of the body, as is the case with cervical cancer. Although technological advances have been made in recent years, gene expression profiling continues to be a prominent approach in the investigation of cervical cancer. Since then, researchers have had the opportunity to examine a gene coexpression network, which has evolved into an exceptionally comprehensive technique for microarray research. This has helped them to get a better understanding of the human genome. When a specific biological issue is addressed, gene coexpression networks retain a considerable percentage of their once vast component of physiognomy, which was previously immense. When comparing the properties of genes in a population, it is well known that feature selection may be used to choose genes that outperform the rest of the genes in the population. There are several benefits to feature selection, and this is only one of them. Typically used gene selection approaches have been shown to be insufficient in acquiring the best potential sequence of genes for training purposes, and as a result, the accuracy of the classifier has likely suffered as a result of this. Recently, a considerable number of scientists have advocated for the use of optimization approaches in the process of gene selection, and this trend is expected to continue. A metaheuristic algorithm may be used to choose a suitable subset of genes, according to the preceding assertion, which is also consistent with the metaheuristic approach. A Modified Probabilistic Neural Network differs from other networks in that the underlying gene expression associated with DEGs and standard data in a Modified Probabilistic Neural Network is not uniformly distributed as it is in other networks (MPN). As previously said, selecting the most relevant genes or repeating genes is a vital step in the prediction process. It was this technique that was used in the research of cervical cancer. Since then, researchers have had the opportunity to examine a gene coexpression network, which has evolved into an exceptionally comprehensive technique for microarray research. This has helped them to get a better understanding of the human genome. When a specific biological issue is addressed, gene coexpression networks are able to preserve a previously major section of the face that had been lost. When comparing the properties of genes in a population, it is well known that feature selection may be used to choose genes that outperform the rest of the genes in the population. There are several benefits to feature selection, and this is only one of them. Typically used gene selection approaches have been shown to be insufficient in acquiring the best potential sequence of genes for training purposes, and as a result, the accuracy of the classifier has likely suffered as a result of this. In the field of gene selection, several scholars have argued in favor of the employment of optimization approaches. A metaheuristic algorithm may be used to choose a suitable subset of genes, according to the preceding assertion, which is also consistent with the metaheuristic approach. It was discovered that Modified Probabilistic Neural Networks (MPNs) had a different distribution of gene expression linked with DEGs and normal data than other networks, which had not been previously seen. This was previously unknown. Following what has been said before, selecting the most appropriate or repeated genes is a critical task throughout the prediction process.

## 1. Introduction

For IA1 individuals, a local procedure such as conization or a full hysterectomy is recommended, depending on the patient's desire to remain fertile. Patients with IA2 are advised to undergo a radical operation such as a pelvic lymphadenectomy if they want to maintain their reproductive potential. Approximately 8% of individuals have lymph nodes in the pelvis that are positive for the disease on average. At this stage of the disease, radical trachelectomy is becoming a feasible option for these women in order to preserve as many of their reproductive options as possible. Individuals suffering from IB1 may also benefit from the same therapy. A combination of intermediate-risk factors (vascular and lymphatic permeation, tumour size greater than 2 cm, deep cervical stromal invasion, and positive surgical margins) or high-risk factors (positive pelvic lymph nodes, parametrial infiltration, and positive surgical margins) is present in early cases that are surgically treated. In most circumstances, individuals with early-stage cancer have a fair prognosis, with 5-year survival rates above 90 percent in the vast majority of cases.

Women in industrialized countries die from cervical cancer at a higher rate than women in developing countries, according to the World Health Organization [1]. One of the most frequent malignancies globally, hepatocellular carcinoma (HCC), has the greatest effect in developing countries such as India and China, where the illness has the greatest impact. Using a genetic approach to cervical cancer, researchers hope to uncover particular essential genes that are involved in the course of the disease. This is an emerging technology that is becoming more important. Tumors, such as cervical cancer, spread via the accumulation of genetic defects that accumulate over time, as is the case with all malignancies, and this is especially true for cervical cancer. This process is referred to as carcinogenesis in medical terminology. As a result of this revelation, it is likely that a better knowledge of the condition and, therefore, more effective treatment options [2] may become available. In conjunction with statistical techniques, gene expression patterns have been used to explore a diverse range of malignancies, including breast cancer [3, 4].

Because of the present interest in biological networks and because of the current interest in biological networks, a gene coexpression network has been developed as a new universal technique for microarray analysis in accordance with the current interest in biological networks (GCEN). This method allows researchers to monitor the expression levels of thousands of genes, or even the whole genome, in a single experiment, allowing them to conduct several experiments in one setting. A higher dataset is required to achieve higher accuracy in computational intelligence. In order to take use of this potential, gene coexpression networks have been frequently employed to widen the scope of biological research to include the whole genome, which has shown to be very beneficial. The differential expression analysis (DCA) approach is being developed as a distinct complement to standard differential expression analysis [4] when two genes coexpress in a differentiating mode of expression, in addition to the more traditional way of differential expression analysis.

According to what has already been shown, many of these traits, on the other hand, are inapplicable when investigating a particular biological state that is not in dispute. It follows as a result that, when choosing a limited subset of genes with the purpose of boosting the output of experiments that are primarily focused on this restricted subset of genes, careful feature selection is necessary. Given the fact that standard feature selection techniques are unlikely to provide the most comprehensive set of features conceivable, it is likely that the performance of a classifier would suffer as a consequence of this shortcoming. The use of optimization techniques has become more popular among researchers in order to help them in selecting the qualities that they want to use in their investigations. Part of the proposed research includes the introduction of a feature selection strategy based on the metaheuristic algorithm [5], which is used as an optimal search tool to choose a subset of characteristics from a larger range of characteristics.

Normalization of the gene dataset is essential in order to guarantee that aspects of the gene dataset that are not significant to the gene dataset are removed from the gene dataset. This goal is achieved by the use of the fuzzy C Means (FCM) technique for modelling. Using tests, it has been shown that coupling the suggested IBO with the SVM approach leads to enhanced accuracy in classifying performance for the gene expression datasets that have been provided.

## 2. Methodology

In order to get the best gene selection and classification outcomes in cervical cancer, it is advised that the Improved Bat Optimization (IBO) approach be utilized in combination with the Support Vector Machine (SVM) method. The suggested technique's structure includes steps for data standardization, [6] module identification, gene selection, and classification, all of which are important for the method to be successful. At a high level of abstraction, the model that has been given is shown in Figure 1.

### 2.1. Normalizing Gene Data Using FCM

Cervical biopsy samples from patients who had been diagnosed with cervical cancer were used in the study. A written informed consent was obtained from each participant prior to the collection of the samples in question, in accordance with the Kasturba Hospital's ethical committee. DNA was acquired from a variety of sources, including tissue biopsy, Pap smear, and cell lines, among others. To prepare the biopsy samples, they were washed and diced into small pieces, which were then put on sterile Petri dishes using sterile 1XTBS solution. Afterward, it was placed in a 1.5-mL microcentrifuge tube filled with 500 L DNA extraction buffer (50 mg Tris pH 8.0, 200 mg NaCl, 20 mg EDTA pH 8.0, and 1 percent SDS) and centrifuged for 15 minutes at 1,500 rpm. In order to get the RNAse product, the lysate was transferred to a 1.5 mL microcentrifuge tube and incubated at 37°C overnight with 10 g/mL proteinase K and 10 g/mL RNAse. The tube was inverted a few times throughout the experiment to guarantee that it did not create a vortex at any point over the duration of the experiment. Following the completion of the digestion procedure, about equal amounts of buffer saturated phenol were added to the 1.5 mL microcentrifuge tube and stirred for 20 minutes.

Afterward, the contents of the tube were centrifuged at 12,000 rpm for 15 minutes at 4°C, following which they were thrown away.

Removed from the tube and transferred to a new tube, the top layer was a result of the procedure. The reaction was terminated after 15 minutes of mixing at room temperature with equal parts chloroform and isoamyl alcohol (24 : 1), according to the protocol. It was necessary to spin the tube a second time at 12,000 rpm for 15 minutes at 4°C, after which the top layer was transferred to a sterile 1.5 mL microcentrifuge tube for use in the next step. To this, 1/10th volume of 3 M sodium acetate was added, along with twice the amount of 100 percent ethanol, and the combination was allowed to settle at −80°C for 2 hours before being discarded. The tube was centrifuged at 12,000 rpm for 15 minutes at 4°C, and the supernatant was removed after the centrifugation at 12,000 rpm. In order to extract the pellet from the mold, 500 mL of 70 percent ethanol was poured over it. The tube was centrifuged in the same way as before, and the supernatant was removed and disposed of as before. It was necessary to dry the tubes on a bench top until they were semidry before putting them away. This was then mixed with about 50 mL of 1XTE pH 8.0 (10 mM Tris/1 mM EDTA Buffer) or MilliQ water, which was left to rest on the bench until completely dissolved before using. The DNA was then stored at −20°C until it could be repurposed in another experiment. A total of 500 mL of DNA extraction buffer was added to the cells after they had been washed twice with PBS and centrifuged at 800 rpm for 5 minutes. This allowed us to get DNA from cell lines and exfoliated cells separately. Similar to the procedures used for DNA extraction from biopsy samples, the following steps in the procedure were followed for DNA extraction from blood samples.

A user's input is normalized and missing values are filled in before any information is shown to them. This is done before any information is displayed to them. The raw data are normalized by using the log-ratio (median of CHI/CH2) as a criterion for the raw data and calculating the resulting standard deviation. Using the example of residual genes, the data gaps were filled in by computing the mean value of the remaining samples taken under comparable conditions in the lab. To replace the probe sets that had previously been employed, a clustering strategy is used in conjunction with other techniques. The purpose of clustering analysis is to produce partitions of gene data that are based on the similarity of the gene information contained in the data set rather than the similarity of the genes themselves. When data is partitioned, it is separated into a large number of clusters, which is represented by the fuzzy partition matrix *U*, which is shortened as fuzzy partition matrix *U*. The membership values *ij* for each gene *I* in each cluster *j*, as well as the membership values *ij* for all genes in all clusters, are included in this collection of membership values. It is possible to characterize the fuzzy partitioning space *M*_*fc*_ with relation *R* as follows, using the following equation:

(1) $$\begin{array}{c} \left.\begin{array}{cc} M_{fc}=\left\{U_{j}\in R^{c\times N}|\right. & \sum_{i=1}^{c}\mu_{ij}\left\{0,1\right\}\forall i,j\\ 0<\sum_{j=1}^{N}\mu_{ij}<N\forall i \end{array}\right\}. \end{array}$$

Here, *c* represents the number of clusters, and *N* represents the entire amount of genetic information. As explained further below, a critical objective function for fuzzy clustering [7] is the c-means functional Jm, which weights the summation of squared errors inside the clusters based on the c-means functional Jm. Gene expression data may be expressed in the following ways, according to the scientific community:

(2) $$\begin{array}{c} \underline{G}\left(G,U,P\right)=\sum \sum {\left(\mu_{ij}\right)}^{m}\left\|g_{i}-p_{j}\right\|A, \end{array}$$

(3) $$\begin{array}{c} \mu_{ij}=\frac{1}{\sum_{i=1}^{c}\left(\left\|g_{i}-p_{j}\right\|A^{\left(2/m-1\right)}/\left\|\theta \right\|A\right)},\;\forall i,j, \end{array}$$

(4) $$\begin{array}{c} p_{j}=\frac{\overset{N}{\sum }{\left(\mu_{ij}\right)}^{m}g_{i}}{\overset{N}{\sum }{\left(\mu_{ij}\right)}^{m-}},\;\forall j. \end{array}$$

Iteration switching between equations (3) and (4) is used to adjust *ij* and *pj* until the variance in Jm falls below a specific threshold or the maximum number of iterations *t* is achieved after a specified number of iterations. The symbol *pj* represents the weighted mean of the cluster *j* data set. It is governed by the fuzzification parameter *m* how fuzzy the partitioning is, or how much gene membership is spread amongst the clusters, and how many genes are in each cluster. With respect to *m* 1, the data's fuzzy clustering converts into the data's hard clustering, as seen in Figure 1. After then, the prototypes pj are nothing more than a technique by which the clusters *j* work, and they are no longer relevant. Each cluster is given a gene I [8] in the same way as the others. The study goes into further detail about this phenomenon and gives advice for how to best utilize the parameter *m* in your calculations. As a distance, the standard Euclidean norm may be established by applying the matrix “*A*,” which is the equivalence matrix of the identity matrix.

WGCNA is being used to design a gene network, which is currently under development.

A commonly used data mining technique for undertaking biological network studies, Weighted Correlation Network Analysis (WGCNA) [9], is based on duo correlations between distinct genetic variables [10]. In addition to module identification, network building, and topological property calculations, it also offers features for gene selection, data display, data simulation, and interfacing with other programs.

A genetic network's nodes are often represented by genes, proteins, or transcripts, but the edges of a biological network are more likely to reflect experimentally discovered commonalities or functional correlations between the nodes and edges of the network. Through the use of network analysis, it is possible to determine the position of a biological entity in relation to its immediate surroundings throughout the network as a whole, allowing for more in-depth investigation. A beneficial use of the notion of converting gene expression data into a network graph that is based on correlation measurements is the discovery of genes that are expressed in a manner that is similar to one another.

It is feasible to use one of a variety of statistical methodologies to determine the degree to which individual expression patterns are comparable to one another. Using a predetermined technique for measuring correlation as well as a specified threshold for each transcript, networks are formed by linking transcripts together with edges that generate some amount of coexpression. When it comes to genetic analysis, the emphasis is mostly on discovering statistical changes among groupings of sample genes rather than on individual genes. A number of explorative clustering algorithms [11, 12] make use of it to partition data into groups of genes with expression patterns that are similar to one another. In order to be successful, the network model for data analysis must be used in conjunction with a correlation measure that reveals similarities between gene expression patterns, and create gene networks necessitates the use of bioinformatic skills in order to properly organize, integrate, assess, and effectively utilize the data. This is necessary in order to generate biological intuitions, which necessitates the use of bioinformatic abilities.

If you are working with CC Gene Data, you may use PAM-DTC to detect module differences.

A method called Partition Around Medoids (PAM) is introduced in this study, which translates a distance matrix into a set of clusters with a predetermined number of clusters. The technique is then applied to the training set in order to identify the proper set of *k*-medoids from among the *k* clusters [12], and the results are reported. In the form of Pearson correlations, which are applied to gene pairings that are differentially expressed, this information is made available. The Pearson correlation coefficient is used to assess the difference in expression levels between each gene pair. Regarding the proposed model, the correlation threshold has been fixed at 0.8 for the sake of simplicity. It is common practise to link together gene pairs that have a correlation bigger than some predetermined threshold when creating differential coexpression networks. Following this limitation led to the production of two DCNs that could be classified into two unique states: the normal state and the abnormal state, respectively.

Unique dynamic branch cutting techniques for finding the proper clusters in a dendrogram based on their morphology were described in Dynamic Tree Cut [13], which aimed to enhance cluster identification by introducing novel dynamic branch cutting algorithms. PAM is being employed in this work for the goal of effective module detection, which is being accomplished via the utilization of cervical cancer gene data. The fixed height cut process, which has a predefined cut height that is generally greater than the cut height using dendrogram, is called first in this technique, and it is followed by the dendrogram cut process, which is called second. It results in the formation of a starting set of gigantic clusters, which are subsequently dispersed into smaller clusters as a consequence of the subsequent processing. It is necessary to distinguish between the ordered dendrogram of each starting cluster and the remainder of the cluster. As a consequence, a collection of cluster-based dendrograms is produced, which are denoted by the letters H1, H2, and so forth. Following that, PAM runs over each cluster and processes it [14]. While the procedure is in progress, new clusters are produced, and the value of “” is updated to reflect the most recent clusters that have been added to the database. In addition, PAM is called for each and every cluster in the system. This procedure is repeated continuously until there are no new clusters generated in the system. Using the distance metric Bhat that is described in PAM, clustering may be accomplished [15]. In addition, the medoids serve as great representations of the positions of the cluster centers they represent. They are particularly remarkable in light of the fact that a large number of components do not become the property of any one cluster of elements in the aggregate. Because of the user's existing understanding of gene expression data clustering and partitioning, PAM may uncover both small clusters and excellent partitions around medoids in a relatively short period of time. When the number of criteria for producing similarity genes is increased, PAM may be utilized to manufacture them more expertly and effectively [16].

It was feasible to estimate the similarity between a pair of genes by using the adjacency function, which then allowed researchers to calculate the distance between them. The name “Pearson” refers to the correlation function that is utilized. Initially, it begins with a basic set of medoids and then iteratively substitutes one gene among the medoids and one gene among the nonmedoids, starting with the medoids.

When it does, the overall distance between the clusters that are formed as a consequence of it grows. It creates a random selection of *k* representative medoid data bits from a large pool of available data. The total switching cost S is determined for every pair of nonmedoid data items *x* and a chosen medoid *m* that is replaced by *x* when *S* equals or exceeds zero. Switching costs are zero if *S* is larger than zero, and else they are zero. Following that, every residual data item is allocated to a cluster depending on how similar the item in question is to the normal medoid. This process is repeated for every residual data item. The medoids should be checked as often as required until no change is seen.

### 2.2. PAM-DTC

1. To define the clusters, descriptors derived from the data set should be used to describe the genes.
2. Select *k* sample products to be used as medoids at random from the list.
3. Determine the total switching cost *S* for each pair of nonmedoid data *xi* and each pair of medoid *mk* with the use of the following formula: (*ximk*). As long as *S* is less than zero, *mk* is switched with *xi* for each pair of *xi* and *mk* that exists. Assign each data item to the cluster that includes the representative item that is the most similar to the data item in question, commonly known as the medoid cluster.
4. Repeat steps 2-3 as many times as required until there is no change in the medoids' appearance or function.
5. Recognizing clusters in the form of a dendrogram (tree of life diagram).
6. Using the gene dataset that has been provided to you, create the most informative modules that you can.

It is more appropriate to consider the filtered genes as nodes in the network rather than as nodes in and of themselves when creating the coexpression networks. Those gene pairs that are more similar than a certain threshold are linked together, and a DCN may subsequently be created in the manner envisioned by the programmer based on this information.

The network depicts the link between various levels of gene expression data collected over a period of time. In the case of the link between the levels of two expressed genes that has been found, Single Nucleotide Polymorphisms (SNPs) may account for at least a portion of this association at least in part. In gene network reconstruction, it is critical to have connected gene expression properties because genes that are strongly correlated are more likely to have comparable activities, a point that has been underlined before.

#### 2.2.1. HSIC-IBO Model for Gene Selection

If the kernel of *y* is considered to be *B*, then dependency between the exposures and dependence between the *y* used as the response variable is calculated [17] by empirical HSIC in the following way:

The root of tr(HKHB) Equals the root of tr(HXTuuTx HB) (5).

With an increase in the size of *u*, the goal function (5) grows to an arbitrarily large magnitude [18]. The need for sparsity while constraining the length of *u* to a single length is required in order to accomplish the feature selection assignment. The ideal solution is discovered via the application of a method known as the bat algorithm.

When using the bat algorithm in [19], we are attempting to emulate the echolocation behavior of bats [21]. They come in a range of sizes, styles, and colours to suit your needs. Regardless of their size and weight, all bats display very identical behavior whether traveling, hunting, or diving in water [21], regardless of their species. Microscopic bats, for instance, make considerable use of their echolocation ability. While searching for prey or avoiding threats in full darkness, this feature is very beneficial to microbats' survival. Consider Microbat's behavior from the perspective of a fresh optimization method in order to better comprehend it [22]. The bat technique may traverse the search space using position and velocity vectors (or updated position vectors) in order to locate a collection of genes from coexpression networks that were of interest to the user. Every bat in a d-dimensional search space has a frequency (*Fr*), a position (*gf*_*i*_), and a velocity (*Ve*_*i*_) that correspond to a frequency (*Fr*) and a location (*gf*_*i*_) corresponding to a frequency (*Fr*) and a location (*gf*_*i*_) (*gf*_*i*_). In this chapter, the vectors of position, velocity, and frequency are introduced and discussed.

(5) $$\begin{array}{c} V\left(t+1\right)=Ve_{i}\left(t\right)+\left(gf_{i}\left(t\right)-\text{Gbest}\right)Fr_{i},\\ g\left(t+1\right)=gf_{i}\left(t\right)+Ve_{i}\left(t+1\right). \end{array}$$

*Pseudo Code: A. Parameters*: The following parameters are used to solve the problem.

  Bat Population: Gene Pulse Frequency: Features
  Pulse Rate: Gene feature rate Loudness: Irrelevant feature.
  Velocity: Moving from one gene to another.
  Positions: Number of genes.

#### 2.2.2. Topological Relation between Gene Samples

*(1) Pseudo code: Support Vector Machine (SVM)*. Given cancer dataset CD = (sg_1_, *y*_1_),…, (sg_*n*_, *y*_*n*_), Cs//sg_*i*_, *y* are samples with labels, Cs-class [11] (Algorithm 1).

Categorize the genes as cancer and noncancer.

### 2.3. Experimental Results

To appraise the performance of the imposed models, initially, the experiment is performed by utilizing gene data. Cervical cancer microarray samples are collected from GEO (https://www.ncbi.nlm.nih.gov/GEO/). Moreover, the results of the classifiers are implemented using the MATLAB environment [23].

#### 2.3.1. Dataset Description

Specifically, the gene data in the GSM99077 dataset has been separated into two phases of the channel, referred to as CH1 and CH2, and each phase has been labeled with a Cy5 or a Cy3 label, as appropriate. Chromatin homogenate (CH1) is composed of cervical cancer tissue obtained by biopsy of a tumor stage IIIB and total RNA extracted from the tissue sample [24]. CH2 is made out of a normal (nonmalignant) cervical tissue sample obtained from a radical hysterectomy and extracted from total RNA, which is then used to make a vaccine. A total of 54 characteristics are available for each gene dataset, from which combinations of fluorescence intensity mean and median, background fluorescence intensity mean and median, a sum of medians and means and their ratio, as well as a sum of medians, means, and their ratio, are selected for experimental findings [21].

Specifically, the gene data in the GSM99078 dataset has been separated into two phases of the channel, referred to as CH1 and CH2, and each phase has been labeled with a Cy5 or a Cy3 label, as appropriate. It was necessary to extract the RNA from normal (nonmalignant) cervical tissue obtained through a radical hysterectomy and add it to CH1 in order for it to be useful. CH2 was created using RNA extracted from ten distinct human cell types. Cell lines from adenocarcinoma, mammary gland Melanoma, hepatoblastoma, liver liposarcoma adenocarcinoma, cervix histiocytic lymphoma, macrophage, histocyte, and several other types were used in this study. The number of features and their descriptions in the first dataset, GSM99077, and the second dataset, GSM99078, are the same as in the first and second datasets, respectively. They are used in the third and fourth chapters of the book [19] as well as in the introduction.

Four unique phases of cervical cancer with IB1, IA2, IIA, and IB2 are represented among the 300 samples of recurrence genes in the GSE44001 dataset. The largest diameter, disease-free survival (dfs months), and the status of disease-free survival were extracted from total RNA using the Cy3 label. This dataset has been connected with the GPL14951 platform ID for identification purposes. This dataset is being utilized in the proposed work in Section 5and has already been made available.

#### 2.3.2. Evaluation Measure for Proposed System

*(1) Precision and Recall*. Recall, also named as sensitivity, is computed by true-positive rate, whereas precision is computed with Predicted Positive Value (PPV) [3].

(6) $$\begin{array}{c} \text{Precision}\left(\text{Pr}\right)=\frac{\text{tpv}}{\left(\text{tpv}+\text{fpv}\right)},\\ \text{Recall}\left(\text{Re}\right)=\frac{\text{tpv}}{\left(\text{tpv}+\text{fnv}\right)}. \end{array}$$

*(2) The Area under the ROC Curve*.  Table 1 shows the performance metrics of the proposed work. In order to demonstrate the diagnostic capabilities of a binary classifier system when the discrimination threshold of the system is modified [5], Receiver Operating Characteristic (ROC) curves are plotted against the threshold value. The ROC curve may be produced and examined when the TPR and the FPR are plotted against each other at different threshold values [8, 25]. Here Table 1 gives the Performance analysis via False-Positive Rate vs. True-Positive Rate. Although IBO-SVM is the preferred classification algorithm, as illustrated in Figure 2, the average value of the ROC curve for the other classification algorithms, such as DCA and DCN, is 76.5 percent and 86.3 percent, respectively, for the other classification algorithms, according to the preferred classification algorithm, according to the preferred classification algorithm (IBO-SVM). When the suggested model is compared to the other models, it becomes clear that the recommended model's distinguishing efficiency is much larger than that of the others [25]. Here Table 1 gives the Performance analysis.

Figure 3 depicts the results of the ROC curve analysis for three algorithms, including DCN, DCA, and IBO-SVM. The results are separated into three parts, and each section is divided into three portions. Also shown is that the suggested IBO-SVM approach has a higher TPR, ranging between 0.9 and 1, when compared to other models, such as the DCA, which yield TPR rates between 0.8 and 0.9 and between 0.75 and 0.8, respectively (see Figure 3).

#### 2.3.3. Classification Results

In the suggested research, a new model, the IBO-SVM, surpasses variant models when it comes to accuracy [26]. The performance of the classifier is tested using the multiple performance measures described above, and all of the assessments are carried out using both normal and malignant datasets, which produces superior results when compared to the presently existing methodologies in the field [27].

Table 2 shows the recommended model outperforms DCA in terms of precision, sensitivity/recall, F-measure, specificity, and accuracy, while DCA outperforms DCN in terms of precision, sensitivity, F-measure, specificity, and accuracy [28].

Using the cervical cancer dataset as an example, Figure 2 displays a comparison of three different classifiers using a precision metric for the cervical cancer dataset [29]. The number of processes is indicated by the *x*-axis, and the metric values are represented by the *y*-axis in this diagram. In the experiments, it was discovered that the supplied IBO-SVM technique obtains a better accuracy value of 91.59 percent, which is 1.84 percent and 0.65 percent higher than the DCA and DCN methods, respectively, and that the algorithm is more efficient than the other approaches [30].

Figure 4 shows the recall comparison of the cervical cancer dataset using three different classifiers shown in the following image. As shown by the experimental results, the proposed IBO-SVM algorithm has a higher recall value of 90.66 percent, which is 20.66 percent and 14 percent greater than the DCA and DCN algorithms, respectively, and is thus preferred [31]. Figure 4 shows the recall comparison of the proposed work.

As seen in Figure 5, the f-measure comparison of classification algorithms was performed [32]. The number of classifiers is indicated on the *x*-axis, while the f-measure values are depicted on the *y*-axis in the graph below. Researchers discovered that the f-measure value obtained using the proposed IBO-SVM algorithm is 91.13 percent, which is 10.21 percent higher than the DCA technique and 5.22 percent higher than the DCN approach, based on their results [33].

On the right-hand side of Figure 6, you can see a comparison of specificity across various classification algorithms. The proposed IBO-SVM method outperforms both the DCA and DCN processes in terms of specificity, achieving a value of 90.50 percent, which is 21.05 percent greater and 14.89 percent higher, respectively, than the other two techniques [34].

Figure 7 shows the accuracy evaluation for the cervical cancer dataset for the purpose of demonstration. Specifically, when compared to the DCA and DCN approaches, which were previously discussed in Table 2, the experimental results reveal that the proposed IBO-SVM algorithm achieves a higher accuracy value of 91.56 percent, which is 8.06 percent and 4.81 percent, respectively, higher than the DCA and DCN approaches [35].

In order to separate curcuminoids, thin-layer chromatography (TLC) was utilized, and the Rf values for curcuminoids from C, DMC, and BDMC were, respectively, 0.75, 0.55, and 0.27 for curcuminoids from C, DMC, and BDMC [36]. With the enhanced resolution of the Rf value, it was established that chloroform and methanol could be utilized as solvents in column chromatography for the separation and separation of diverse compounds [37]. When Gupta et al. explored alternative compositions of the mobile phase for the separation of curcuminoids, it was revealed that utilizing chloroform and methanol (95 : 5) as the mobile phase allowed them to accomplish the necessary separation. The Rf values found for C, DMC, and BDMC were 0.69, 0.44, and 0.29, respectively, with C being the most favorable. During the separation column chromatography process, a continuous difference in Rf value is critical to the success of the procedure [38].

In column chromatography, separation is accomplished by elution with chloroform and methanol, with the polarity of the elution solutions increasing as the separation proceeds [39]. UV spectroscopy was used to determine the total curcuminoids present in the fractions, which were found to be 84 percent, 86 percent, 80.6 percent, and 80.6 percent of C, DMC, and BDMC, respectively, in the fractions. A few fractions showed two distinct curcuminoids in TLC due to the 10–15 percent loss of curcuminoids that occurred during the extraction process; as a consequence, they were concentrated and chromatographed on the column for further separation [40]. It is estimated that 8.8 percent of the pigments were wasted on average due to the difficulty of separating colors mixed together on the column. Following the completion of further purification, the following products were obtained: curcumin crystals that are bright yellow needle-shaped, DMC crystals that are light yellow, and BDMC crystals that are reddish-orange in color.

## 3. Conclusion

Using the IBO-SVM methodology to determine the gene expression profile of microarrays is addressed in detail in this chapter, as well as how it varies from other approaches. A unique swarm-based strategy known as IBO gene selection has been developed with the goal of picking the most informative genes from among a large number of potential candidates. As a result, it is employed in the resolution of cervical cancer classification paradigms that deal with high-dimensional information, such as microarray gene expression profiles, and in enhancing the overall accuracy of the classification system. An optimum gene selection in a microarray dataset may be achieved using the HSIC strategy, which picks genes from a sample in order to get the highest number of genes feasible. Applying the IBO-SVM technique presented in this paper to a microarray dataset, the goal is to identify the gene with features that are both similar and instructive in nature. In addition, the SVM classifier is trained and evaluated, with the classification accuracy being tested using the genes that have been selected for inclusion in the analysis. In this study, it was discovered that although the proposed technique gives higher classification results for gene-gene expression datasets, it continues to present difficulty for datasets with uneven distributions of gene expression levels.

## Figures and Tables

**Figure 1:** Flowchart of the proposed system.

**Figure 2:** Precision comparison vs. classifiers.

**Figure 3:** Area under ROC curve vs. three models.

**Figure 4:** Recall comparison vs. classifiers.

**Figure 5:** F-measure results comparison vs. classifiers.

**Figure 6:** Specificity results comparison vs. classifiers.

**Figure 7:** Accuracy results from comparison vs. classifiers.

**Algorithm 1:** Pseudo code of PNN.

**Table 1:** False-positive rate vs true-positive rate.

FPR	TPR		
	DCA	DCN	IBO-SVM
0.02	0.72	0.83	0.93
0.04	0.76	0.86	0.95
0.06	0.77	0.865	0.965
0.08	0.783	0.870	0.98
1	0.790	0.890	1

**Table 2:** Performance comparison analysis.

Methods	Precision (%)	Recall (%)	F-measure (%)	Specificity (%)	Accuracy (%)
DCA	89.75	70	80.92	69.45	83.50
DCN	90.94	76.66	85.91	75.61	86.75
IBO-SVM	91.59	90.66	91.13	90.5	91.56

## Data Availability

The data sets used are available at https://www.kaggle.com/competitions/cervical-cancer-screening/data.
